RETRACTED

# si-PDGFR*β*-Loaded Exosomes Suppress the Progression of Glioma by Inhibiting the Oxidative Associated PI3K/Akt/EZH2 Signaling Pathway

**DOI:** 10.1155/2022/5081439

**Published:** 2022-10-14

**Authors:** Yuping Li, Hailong Yu, Qiang Ma, Min Wei, Xiaoguang Liu, Yajie Qi, Chen Li, Lun Dong, Hengzhu Zhang

**Affiliations:** ^1^Neuro Intensive Care Unit, Clinical Medical College, Yangzhou University, Yangzhou, China; ^2^Department of Neurosurgery, Clinical Medical College, Yangzhou University, Yangzhou, China; ^3^Department of Neurosurgery, Changzhou No. 2 People's Hospital, Changzhou, Jiangsu, China

## Abstract

This study investigated the possibility of exosomes loaded with si-PDGFR*β* ability to suppress the progression of glioma. Common gliomas develop from neuroglial progenitor cells. Many variables affect the survival rate and occurrence of gliomas. Understanding oxidative stress processes and creating new, efficient treatments are crucial because oxidative stress is linked to the development of brain tumors. For this purpose, selected clinical samples were subjected to various tests like quantitative real-time PCR, Cignal Finder RTK signaling 7-pathway reporter array analysis, CCK-8 analysis, flow cytometry, and immunoblotting. Here, we demonstrated that PDGFR*β* expression was increased in glioma patients. Following that, cell-derived exosomes were extracted and collected and traced *in vivo,* and selected tissue samples were subjected to immunohistochemical analysis. The results indicated that the knockdown of PDGFR*β* (si-PDGFR*β*) inhibited the proliferation of glioma cells. Besides this, si-PDGFR*β*-loaded exosomes induced a similar antitumor effect in glioma cells. The anticancer effect of si-PDGFR*β*-loaded exosomes was mediated by the inactivation of the PI3K/Akt/EZH2 pathway. Finally, we verified that this exosome delivery system, si-PDGFR*β*-loaded exosomes, had robust targeting and no associated toxicity. In conclusion, the study confirmed that si-PDGFR*β*-loaded exosomes inhibit glioma progression via inactivating the PI3K/Akt/EZH2 signaling pathway.

## 1. Introduction

As the most common central nervous system (CNS) tumor, glioma accounts for over 26.6% of all CNS tumors, among which glioblastoma (GBM, WHO grade IV) with a low five-year survival rate (about 5.5%) occupies approximately 56.1% of all gliomas [1, 2]. The imbalance between oxidative and antioxidant activity in the body is referred to as oxidative stress. As part of regular metabolism, oxygen is reduced by electrons, creating numerous reactive oxygen species (ROS). The main contributors to oxidative stress are ROS, which can be directly detected and quantified. In addition to having defensive mechanisms that aid in the elimination of bacteria and pathogens, oxidative stress has the potential to damage host cells through increased ROS accumulation. One of the most prevalent malignant tumors of the central nervous system is glioma, distinguished by redox state alterations. Even low-grade glioma with a good prognosis (including LGG, WHO grade I or II) inevitably relapses and develops into high-grade glioma (such as HGG, WHO grade III or IV) [3]. The abnormal proliferation, high invasion ability, high tolerance to hypoxia, existence of cancer stem cells, and immune escape from the microenvironment in GBM tumors cause therapeutic failure and adverse prognosis. For patients with GBM, the median overall survival time is only 14.5 to 16.6 months, even with aggressive surgical treatment combined with postoperative chemoradiotherapy [4]. Consequently, it is important to search for biomarkers of diagnosis and prognosis for the early diagnosis and progression detection of glioma and to improve the treatment efficiency.

RETRACTED

The PDGF family's five subtypes regulate various cellular functions, such as proliferation, differentiation, and activation of signal transduction, by binding to two specific receptors (PDGFR-*α* and PDGFR-*β*) [5]. PDGFR-*β* is an essential promoter of cell division and a vital polypeptide growth factor [6]. Several studies have confirmed that PDGFR-*β* can preferentially bind with PDGF-BB and have a strong promoting effect on the proliferation and differentiation of cancer cells [7]. For example, missense mutations in the exon of the PDGFR-*β* gene are associated with tumorigenesis and cell proliferation [8]. Furthermore, studies have shown that PDGF-BB and PDGFR-*β* knockout mice have severe cardiovascular and renal dysplasia, accompanied by aortic dilatation and bleeding. It suggests that PDGFR-*β* stimulates tumor angiogenesis by activating adjacent tissue cells and releasing vascular endothelial growth factors [9]. Many inhibitors and proangiogenesis factors determine the formation of tumor angiogenesis, among which PDGF family members are one of the essential factors in tumor angiogenesis [10]. Therefore, antitumor treatment strategies for PDGFR targets are getting more and more attention.

Modulating oxidative stress is considered to be an important method of treating cancer. Many kinds of oxidative medicine have been reported, including small molecule compounds, natural products, and nucleic acid drugs. In recent years, with the gradual deepening of exosome research, it has been gradually found that exosomes also play an important role in regulating cell oxidative damage and ROS. Exosomes are vesicles with a diameter of 30-100 nm [11]. They are secreted by all kinds of cells, including proteins, nucleic acids, and other components, and have been shown to modify the formation of an immunosuppressive tumor microenvironment [12, 13]. Studies have shown that exosomes carry long noncoding RNAs (lncRNAs), mRNAs, and microRNAs (miRNAs) and regulate the biological behavior of target cells by delivering these RNAs to target cells [14]. Therefore, exosomes play a crucial role in material and information exchange between cells. Exosomes are thought to be the carrier of many oncogenic factors and participate in developing glioma. In glioblastoma (GBM), the epidermal growth factor receptor (EGFR) variant III (EGFRv III) and other carcinogenic components are transferred to the microenvironment through exosomes and spread invasiveness [15]. It has been reported that VEGF was transported by glioma-derived exosomes (GEXs) to promote the formation of glioma blood vessels [16]. Exosomes, as a kind of vesicle secreted by cells, have good application potential in drug delivery. Compared to other nanodelivery systems such as lipids, polymers, and gold, live cell-derived exosomes have low immunogenicity. They are highly biocompatible nanocarriers and exhibit greater flexibility and very low cytotoxicity in loading the required antigens for efficient delivery [17, 18].

RETRACTED

Moreover, exosomes do not have the problem of adsorbing proteins to produce protein crowns, which can achieve stable drug transport in the blood. The PI3K/Akt/mTOR signaling pathway is a significant pathway in regulating oxidative stress. Here, we show that exosomes loaded with si-PDGFR*β* derived from pericytes exhibit antitumor properties through retarding the activation of the PI3K/Akt/mTOR signaling pathway in glioma.

## 2. Materials and Method

### 2.1. Clinical Samples

Fifty-nine patients with glioma were randomly selected for this study who were hospitalized in the Neurosurgery Department of Clinical Medical College of Yangzhou University and underwent surgical treatment from Jan 2020 to May 2021. Pathological types were based on WHO neuroepithelial tumor classification criteria. They were divided into the low-grade group (31 cases with WHO grade I-II, 15 males and 16 females) and high-grade group (28 cases with WHO grade III-IV, 16 males and 12 females), and 12 brain tissue resections from traumatic brain injury patients were selected as the control group. The Ethics Committee approved the experiments for the Clinical Medical College of Yangzhou University.

### 2.2. Quantitative Real-Time PCR (qRT-PCR)

Total RNA extraction was performed with TRIzol reagent (AM1912, Thermo Scientific) and evaluated the quantity and purity of RNA with NanoDrop ND-1000 spectrophotometer (Thermo Scientific). Complementary DNAs were synthesized using an invalidated transcription kit (RR037A, Takara) and implemented as models for PCR assay. The Primer Premier 5.0 software was used to create the following primers for this study: PDGFR*β* forward: 5′-ACTGCCCAGACCTAGCAGTG-3′ and reverse: 5′-CAGGGAAGTAAGGTGCCAAC-3′ and GAPDH, forward: 5′-CAG GAGGCATTGCTGATGAT-3′ and reverse: 5′-GAAGGCTGGGGCTCATTT-3′. These primers were synthesized by Sangon Biotech (Shanghai, China).

RETRACTED

### 2.3. Cignal Finder RTK Signaling 7-Pathway Reporter Array

To ascertain the critical downstream pathways regulated by PDGFR*β*, Cignal Finder RTK signaling 7-Pathway Reporter array was performed. Subsequently, the pathway-specific transcription factor or control constructs were transfected into U251 cells. The relative activity of each signal pathway was driven by Dual-Luciferase® Reporter Assay System from Promega (Promega, Beijing, China).

### 2.4. Cell Counting Kit-8 (CCK-8) Assay

U251 cells (1 × 10^4^ per well) were seeded into 96-well plates. At 0, 24 h, 48 h, and 72 h, 10 *μ*L CCK-8 solution was added to each well and incubated with U251 cells at 37°C for 3 hours. U251 cells' absorbance (450 nm) was measured to determine their level of vitality.

### 2.5. Flow Cytometric Analysis (FACS)

Induction of apoptosis in U251 cells was evaluated by PI and Annexin V-EGFP kit (KeyGen Biotech Co., Ltd., Nanjing, China). Briefly, U251 cells (5 × 10^6^ cells/well) were seeded into 6-well plates and collected after transfection with the different plasmids for 48 hours. Finally, these cells were washed with cold PBS at 4°C and analyzed through a flow cytometer.

### 2.6. Immunoblotting

Glioma tissues and cell line (U251) were rinsed with PBS and lysed with RIPA buffer (4693116001, Roche) with a protease inhibitor; the concentrations were examined through a BCA protein assay kit (23227, Thermo Scientific). The total protein sample (30 *μ*g) was separated on 12.5% SDS-PAGE gels and next transferred onto 0.45 *μ*m thin PVDF membranes (Merck Millipore). Blocking with 5% bovine serum albumin at room temperature for 1 hour, membranes were incubated with primary antibodies (as shown in Table 1) at 4°C overnight. After washing, membranes were incubated with secondary antibodies for 1 hour at room temperature. Finally, these protein bands were imaged, contrasted, and analyzed with an ECL assay kit (P0018FS; Beyotime Biotechnology), a ChemiDoc XRS imaging system, and Image Lab software (both Bio-Rad Laboratories, Inc., Hercules, CA, USA), respectively.

### 2.7. Cell Exosome Collection

Conditioned cell culture medium from 1 × 10^7^ pericytes cells cultured for 24 h was collected. The culture media were centrifuged at 800 g for 5 minutes; the supernatant was centrifuged at 2000 × *g*, 4°C, 10 min. Next, the supernatant medium was collected, filtered into a 0.22 *μ*m microporous membrane, and centrifuged at 100,000 × *g*, 4°C for 2 hours. After centrifugation, discard the supernatant, resuspend the tube wall pellet with PBS, and continue to centrifuge for 2 hours at 100,000 × *g* at 4°C. Lastly, after abandoning the supernatant, the exosomal pellet was resuspended in 100 *μ*L PBS and stored at -80°C for subsequent experiments.

RETRACTED

### 2.8. *In Vivo* Exosome Tracing

Exosomes were treated with PKH26 fluorescent dye (2 × 10^6^ M) at room temperature for 20 minutes. This reaction was stopped by 5% bovine serum albumin, resuspended in PBS, and centrifuged (1,500 × *g*, 30 minutes) to separate exosomes. After that, fluorescent-labeled exosomes were injected into rats via tail vein, and perfusion samples were taken after 24 hours of modeling. The exosomes were observed in the tissue sections under a fluorescence microscope to see whether they reached the damaged area. Labeled exosomes were added to pericyte cultures to observe endocytosis under the fluorescence microscope.

### 2.9. Immunohistochemical (IHC) Analysis

For IHC, following deparaffining with xylene and hydration with gradient ethanol, the paraffin-embedded tissue sections were treated with citrate buffer at pH = 6 for 20 min and immersed in a humidified chamber with 3% H_2_O_2_ for 10 min. After washing and blocking, sections were incubated overnight with rabbit PI3K, AKT, and EZH2 antibodies (Table 1) in a humidified chamber at 4°C. Five randomly selected fields were captured using a bright-field microscope (Olympus, Tokyo, Japan) (magnification 200x) and analyzed by Image-Pro Plus v6.2 software (Media Cybernetics, Silver Spring, MD).

### 2.10. Statistical Analysis

Three duplicates of each experiment were carried out. SPSS (version 24; SPSS (IBM) Inc., Illinois, USA) was used for analysis. The classification variants were distributed in numerical numbers. Mean ± standard represented data deviation. Unpaired Student's *t*-test was evaluated for two sets of data comparison, and one-way ANOVA was used for multiple groups. The statistical meaning was determined when *P* < 0.05.

## 3. Results

### 3.1. PDGFR*β* and PDL1 Are Upregulated in the GBM

To interrogate the differential expression of PDGFR*β* in GBM and normal tissues, we integrated GBM data from TCGA and corresponding data of normal brain tissue from the GTEX database. We found that PDGFR*β* in GBM was virtually higher than that in normal brain tissue (Figure S1A). IHC was employed and showed that the expression of PDGFR*β* was higher in GBM than in the adjacent normal tissues (Figure S1B). Then, qrt-PCR results also showed that PDGFR*β* was significantly upregulated in the GBM tissues compared to the normal group (Figure 1(a)). We then compared the mRNA relative expression of PDGFR*β* in glial cells of the human brain (HEB) and four different glioma cell lines (T98G, SHG-44, U251, and HS683) and found that the expression of PDGFR*β* was the highest in U251 cells (Figure 1(b)). According to the qPCR results, PDL1 was also significantly upregulated in the GBM tissues (Figure 1(c)). The expression of PDL1 was notably higher in U251 when compared to HEB cells (Figure 1(d)). Correlation analysis indicated positive results for PDGFR*β* and PDL1 (Figure 1(e)).

RETRACTED

### 3.2. Knockdown of PDGFR*β* Forbids the Proliferation of Glioma Cells

Next, we checked the function of PDGFR*β* on glioma cells naturally. CCK-8 analysis revealed that the cell viability of U251 was virtually diminished by the down-expression of PDGFR*β* (si-PDGFR*β*) (Figure 2(a)). Furthermore, EdU assay results showed that glioma cell proliferation ability was virtually reduced by si-PDGFR*β* (Figure 2(b)). Finally, we tried to analyze whether downregulation of PDGFR*β* could induce apoptosis in the U251 cell line. FACS analysis demonstrated that silencing of PDGFR*β* induced apoptosis in the U251 cell line (Figure 2(c)). Further, immunoblot analysis showed that down-expression of PDGFR*β* significantly boosted the levels of the proapoptotic protein of Bax and cleaved caspase-3 but lowered the level of antiapoptotic protein of Bcl-2 (Figure 2(d)). The above results showed that PDGFR*β* knockdown restrained glioma cell proliferation and induced cell apoptosis.

We then examined the effects of si-PDGFR*β* on glioma cell migration and invasion ability. Wound-healing assay (Figure 2(e)) and transwell assay (Figure 2(f)) showed that PDGFR*β* downregulation inhibited the migration and invasion of glioma cells. Furthermore, down-expression of PDGFR*β* significantly decreased MMP2 and MMP9, the hall marker protein of tumor invasion and metastasis (Figure 2(g)). The above experimental data confirmed that si-PDGFR*β* inhibited glioma cell migration and invasion ability.

### 3.3. Interference with PDGFR*β* Downregulates PI3K/AKT/EZH2 Signal Transduction

We used the Cignal Finder RTK Signaling 7-Pathway Reporter Array to determine which pathways PDGFR*β* regulates to cause downstream gene changes. Overexpression of PDGFR*β* activated the PI3K/AKT pathway, and the knockdown of PDGFR*β* inhibited it (Figure 3(a)). The P85 subunit of phosphoinositide 3-kinase (PI3K) has been reported to bind to phosphorylated PDGFR through the SH2 domain, and serine-threonine protein kinase (Akt) reactivates the downstream molecule. We examined the relationship between PDGFR*β* and PI3K/AKT signaling pathway at the protein level; according to immunoblot analysis, si-PDGFR*β* indeed lowered the levels of p-PI3K and p-AKT proteins (Figure 3(b)). It has been reported that EZH2 promotes tumor occurrence via governing AKT expression [19], and our test results suggested that si-PDGFR*β* significantly downregulated the protein levels of EZH2 (Figure 3(b)). The pattern of PDL1 was also dramatically downregulated by si-PDGFR*β* transfection.

RETRACTED

### 3.4. Identification and Tracing of Exosomes

Transmission electron microscopy (TEM) results showed that the negatively stained exosomes were in the shape of saucers with a diameter of about 100 nm (Figure 4(a)). The particle sizes of exosomes derived from pericytes were concentrated in the range of 80-200 nm, consistent with the consensus of exosome diameter of 30-150 nm (Figure 4(b)). Immunoblot was used to identify exosome molecular markers. The results showed that exosomes derived from pericytes specifically expressed CD63 and TSG101, while the culture medium after exosome extraction did not express such molecules (Figure 4(c)). Exosomes labeled with PKH26 were cocultured with U251 cells, and red fluorescent was observed under a fluorescence microscope as exosomes, indicating that the exosomes could be uptaken by U251 cells (Figure 4(d)). Immunoblots have been applied to identify PDGFR*β* protein expression. The results showed that when exosomes loaded with si-PDGFR*β* were extracted, the protein level of PDGFR*β* in cells decreased significantly (Figure 4(e)).

### 3.5. The Exosomes Loaded with si-PDGFR*β* Resists the Proliferation, Invasion, and Migration of Glioma Cells

Next, we tested whether the exosomes loaded with si-PDGFR*β* exerted tumor inhibition effects in glioma cell lines. The results of the CCK-8 and EdU assays stated clearly that si-PDGFR*β*-loaded exosomes significantly reduced the cell viability of U251 (Figures 5(a) and 5(b)). In addition, FACS analysis revealed that exosomes loaded with si-PDGFR*β* enhanced apoptosis in the U251 cell line (Figure 5(c)). Furthermore, wound healing and transwell assay findings showed that si-PDGFR*β*-loaded exosomes suppressed the invasion and migration of U251 cells (Figures 5(d) and 5(e)).

### 3.6. The Exosomes Loaded with si-PDGFR*β* Exerted Tumor Inhibition Effects on Glioma *In Vivo*

We then explored whether exosomes loaded with si-PDGFR*β* had the same effect in vivo. One week after in situ implantation of glioma cells, PBS, Unloaded-Exo, and si-PDGFR*β*-Exo were injected into tumor-bearing mice via tail vein. Brain MRI was performed on the treated mice after four-week treatment to measure the volume of the transplanted tumor. The results showed that the exosomes loaded with si-PDGFR*β* significantly inhibited the growth of gliomas (Figure 6(a)). We then tested the targeting ability of exosomes loaded with si-PDGFR*β*. We observed that exosomes injected into the tail vein were mainly concentrated at the tumor site through in vivo imaging, suggesting that exosomes loaded with si-PDGFR*β* had relatively high targeting ability (Figure 6(b)). H&E staining indicated that the si-PDGFR*β*-Exo-treated group induced more necrotic cells than the PBS and Unload-Exo groups (Figure 6(c)). TUNEL assay indicated that si-PDGFR*β*-Exo induced more apoptotic cells (Figure 6(c)). The tumor tissue in situ was collected for immunoblot detection. We found that si-PDGFR*β*-Exo significantly decreased p-PI3K, p-AKT, EZH2, and PDL1 proteins, which was consistent with *in vitro* test results (Figure 6(d)).

RETRACTED

### 3.7. *In Vivo* Exosome Treatment Is Safe

We also evaluated the safety of exosome therapy. The body weight was statistically insignificant between the Unload-Exo and si-PDGFR*β*-Exo groups compared with the PBS group (Figure 7(a)). In addition, visceral functional (such as heart, liver, spleen, lung, and kidney) tests showed no statistical difference among these three groups (Figure 7(b)). Also, the biochemical blood test had no remarkable diversities in the liver function of the three groups (Figure 7(c)). Based on the above experimental results, it was suggested that the exosome was safe for treating glioma.

## 4. Discussion

Glioma is a common primary intracranial tumor belonging to the neuroepithelial tumor, which accounts for 44% of intracranial tumors, among which glioblastoma (GBM) with the highest malignant degree, accounts for 22.3% [20]. GBM has the characteristics of strong invasion ability and high malignant degree, and its overall survival rate is still short, even through surgical resection, radiotherapy, and chemotherapy. Oxidative stress is strongly related to the proliferation of cancer cells and is also important in glioma development. Studies have found that GBM is due to the mutation or deletion of tumor suppressor genes and the overexpression of oncogenes, causing cancer cell proliferation and invasion, which are not constrained by normal regulatory mechanisms. Finally, malignant pathological changes occur [21, 22]. Both PDGFR subtypes, PDGFR*α* and PDGFR*β*, are transmembrane glycoproteins whose extracellular N-terminal binding with its ligand activates autophosphorylation of tyrosine residues in the intracellular domain of PDGFR and also activates specific target proteins to promote tyrosine residues phosphorylation, thus transferring the signal into the cell [23]. During embryonic development, PDGFR plays a significant part in physiological activities such as the maturation of the cardiovascular system, connective tissue, central nervous system, gonads, and lungs [5]. PDGFR and its ligands have been proved to be overexpressed in glioma, sarcoma, leukemia, epithelial cell carcinoma, and other malignant tumors and affect the malignant proliferation, vascular hyperplasia, and metastasis of tumor cells. There is a statistically significant positive correlation between PDGFR expression and pathological tumor grade of glioma [24]. Kim et al. have reported that the expression levels of the two receptors were different in glioma. PDGFR*α* was only expressed in a part of GBM patients, while PDGFR*β* expression was more common in GBM patients.

RETRACTED

Moreover, gene therapy targeting PDGFR*β* weakens GBM stem cells' self-renewal and inhibits tumors' proliferation and invasion [25]. In this research, PDGFR*β* expression was remarkably increased in the clinical samples from GBM patients and the U251 cell line. Moreover, consistent with previous studies, knockdown of PDGFR*β* inhibits the metastasis of glioma cells. Moreover, this tumor inhibition was caused by the inhibition of PI3K/AKT/EZH2 signal transduction. Furthermore, we extracted exosomes derived from pericytes and found that exosomes loaded with si-PDGFR*β* have the same tumor inhibition effect. In addition, we have confirmed that this exosome has good safety and targeting properties through experiments and found that si-PDGFR*β*-loaded exosomes inhibited the glioma progression through PI3K/Akt/EZH2 signaling pathway. Besides, PI3K/Akt/EZH2 signaling pathway was upregulated in glioma patients. Collectively, si-PDGFR*β*-loaded exosomes derived from pericytes inhibit glioma's progression via downregulation of the PI3K/AKT/EZH2 signaling pathway.

Exosomes are bioactive nanoscale vesicles secreted by cells and are cup-shaped vesicles with a diameter of 40-140 nm and a lipid bilayer structure [26, 27]. There are many applications for exosomes at present. In the field of diagnosis, Goldie et al. found that among all small RNAs, miRNAs account for a higher proportion in exosomes than in the cells from which they originate [28]. Serum lncRNA HOTAIR can be used as a novel diagnostic and prognostic marker of GBM [29]. The blood-brain barrier (BBB) is one of the significant hurdles in glioma chemotherapeutics. The majority of glioma chemotherapeutic drugs have poor utilization because of their low solubility in blood and short half-life [30]. One of the current technologies used to deliver drugs efficiently and highly targeted to the tumor site is encapsulating drugs in nanocarriers, which often contain targeting factors that facilitate entry into the tumor region [31]. However, the artificial nature of nanocarrier systems leads to problems related to toxicity in vivo. Exosomes, as extensive endogenous carriers, have many favorable drug delivery characteristics: small size, immune escape, the long half-life, and subtypes that target tumor cells [31]. More importantly, exosomes can load hydrophilic and hydrophobic drugs effectively. In this study, exosomes extracted from mouse pericellular cells were observed by TEM to be round or like a tea holder/cup structure, with dark surrounding color and a light center with an obvious three-dimensional sense. The diameter was about 100 nm, and the peak particle size was about 100 nm. The concentration of distribution was high at one time, showing no difference with the characteristics of exosomes previously reported in the literature [12].

RETRACTED

The electroporation method is a mature method to load drugs into isolated exosomes. Its principle is to expose suspensions of exosomes and therapeutic drugs to an electric field, and the exosome membrane will generate numerous holes under a short high-pressure pulse, through which small drug molecules penetrate exosomes [17]. The siRNA is a promising therapeutic solution as a posttranscriptional gene regulation process for various pathological conditions and regulating cellular longevity. Wahlgren et al. measured the loading efficiency with fluorescently labeled siRNA, and the loading efficiency reached 25% [32]. In this paper, si-PDGFR*β* was also transferred into exosomes by electroporation, and exosomes loaded with si-PDGFR*β* had the same tumor inhibition effect as si-PDGFR*β*. Pericytes secrete excessive transmembrane receptors, CD248, and other signal molecules to promote the angiogenesis of gliomas but also guide endothelial cells to secrete vascular endothelial growth factor (VEGF) through the PDGFR*β* signaling pathway synergistically promoting tumor angiogenesis. In addition, endothelial cells secrete more VEGF in high-grade gliomas [33]. We confirmed that the exosomes loaded with si-PDGFR*β* exerted tumor inhibition effects on glioma in vivo and were more robust in targeting low immunogenicity.

PI3K/Akt plays an essential part in the occurrence and progression of malignant tumors and has proven to be one of the therapeutic targets of malignant tumors [34]. Phillips et al. reported that myricetin promoted cell apoptosis in pancreatic cancer by inhibiting the PI3K/Akt signaling pathway [35]. As a polycomb-repressive complex-2 (PRC-2) component, the knockdown of EZH2 gene expression was found to induce cell arrest in the G2-M phase to inhibit cell proliferation [36]. Choi et al. found that EZH2 expression increased in 60.6% of gastric cancer patients but only 6.7% of nonneoplastic patients [37]. The Akt signaling pathway inhibits trimethylation of H3K27 through phosphonate EZH2 and disrupts gene silencing, leading to carcinogenesis [38]. We revealed that exosomes loaded with si-PDGFR*β*, which targeted ZEB1, inhibited glioma cells' invasion, proliferation, and migration via inhibiting the PI3K/Akt/EZH2 pathway. More importantly, *in vivo* experiments revealed that exosomes loaded with si-PDGFR*β* effectively and safely inhibit glioma development.

RETRACTED

## 5. Conclusions

Increased free radical levels and diminished antioxidant defense responses are associated with the development of gliomas. Since oxidative stress plays a significant role in the aetiology of gliomas, antioxidant treatment may be effective in treating tumors. Therapeutic regimens still face numerous difficulties and problems. However, many kinds of oxidative medicine include small molecule compounds, natural products, nucleic acid drugs, and protein drugs. Exosomes, as a favorable carrier for various medicine, including oxidative medicine, could exert their antitumor properties by regulating oxidative stress, which enables their therapeutic effects in inhibiting proliferation and invasion. In summary, *in vivo* and *in vitro* experiments in this study showed that si-PDGFR*β*-loaded exosomes may protect against glioma progression by preventing the activity of the PI3K/Akt/EZH2 signaling pathway. Moreover, evaluate the potential value of exosomes loaded with si-PDGFR*β* as a treatment strategy for glioma.

## Figures and Tables

**Figure 1:** Differential expression of PDGFR*β* in the clinical tissue samples and glioma cell lines. (a) Relative mRNA level of PDGFR*β* in glioma patients (^∗∗^*P* < 0.01 vs. normal group). (b) Relative mRNA level of PDGFR*β* in glioma cells (^∗∗^*P* < 0.01 vs. HEB cell group). (c) Relative mRNA level of PDL1 in glioma patients (^∗∗^*P* < 0.01 vs. normal group). (d) Relative mRNA level of PDL1 in glioma cells (^∗∗^*P* < 0.01 vs. HEB cell group). (e) The relationship between PDGFR*β* and PDL1.

**Figure 2:** The effects of silencing PDGFR*β* on tumor inhibition of U251 cells. (a) U251 cell viability was measured by CCK-8 after transfecting with si-NC or si-PDGFR*β* at 0, 24 h, 48 h, and 72 h. (b) EdU detection showed that si-PDGFR*β* induced apoptosis. (c) FACS analysis showed that si-PDGFR*β* induced apoptosis. (d) Immunoblot analysis showed the levels of the proapoptotic protein of Bax and cleaved caspase-3 and antiapoptotic protein of Bcl-2. (e) Wound healing test showed that si-PDGFR*β* inhibited the migration of glioma cells. (f) Transwell assay results showed that downregulation of PDGFR revealed caspase-cell migration and invasion in glioma. (g) There are indications that si-PDGFR*β* lowered MMP2 and MMP9, the hall marker protein of tumor invasion and metastasis by immunoblot analysis (^∗^*P* < 0.05, ^∗∗^*P* < 0.01, and ^∗∗∗^*P* < 0.001 vs. si-NC group).

RETRACTED

**Figure 3:** The antitumor effects are mediated by knocking down of si-PDGFR-*β* via downregulating PI3K/AKT/EZH2 signaling pathway. (a) The Cignal Finder RTK Signaling 10-Pathway Reporter Array demonstrated that the up-expression of PDGFR*β* activated, and the knockdown of PDGFR*β* downregulated the PI3K/AKT signaling pathway. (b) Immunoblot analysis displayed that down-expression of PDGFR*β* decreased the p-PI3K, p-AKT, EZH2, and PDL1 protein levels (^∗∗∗^*P* < 0.001 vs. si-NC group).

**Figure 4:** Identification of exosomes derived from pericyte. (a) Transmission electron microscopy (TEM) results showed that the negatively stained exosomes were in the shape of saucers with a diameter of about 100 nm. (b) The particle sizes of exosomes derived from pericytes were at about 100 nm according to nanoparticle size analysis. (c) Immunoblot results showed that exosomes derived from pericytes specifically expressed CD63 and TSG101, while the culture medium did not express such molecules after exosome extraction. (d) Red fluorescent was observed under a fluorescence microscope in U251 cells cocultured with PKH26 labeled exosomes. (e) Immunoblot results showed that when exosomes loaded with si-PDGFR*β* were extracted, the protein level of PDGFR*β* in cells decreased significantly (^∗^*P* < 0.05 vs. PBS or Unloaded-Exo group).

**Figure 5:** Exosomes loaded with si-PDGFR*β* resists the proliferation, invasion, and migration of glioma cells. (a) U251 cell viability was measured by CCK-8 analysis after transfected with exosomes loaded with si-PDGFR*β* (si-PDGFR*β*-Exo) at 0, 24 h, 48 h, and 72 h. (b) EdU assay indicated that proliferation ability of glioma cells was significantly reduced by exosomes loaded with si-PDGFR*β*. (c) FACS assay analysis demonstrated that exosomes loaded with si-PDGFR*β* induced more apoptotic cells in the U251 cell line. (d) Wound healing test showed that cell migration of glioma of the si-PDGFR*β*-Exo group was significantly inhibited. (e) Transwell assay results showed that si-PDGFR*β*-Exo inhibited migration and invasion of glioma cells (^∗∗^*P* < 0.01 and ^∗∗∗^*P* < 0.001 vs. PBS or Unloaded-Exo group).

RETRACTED

**Figure 6:** The exosomes loaded with si-PDGFR*β* exerted tumor inhibition effects on glioma *in vivo*. (a) Brain MRI was performed on the treated mice after four-week treatment to measure the volume of the transplanted tumor. The results showed that the exosomes loaded with si-PDGFR*β* significantly inhibited the growth of gliomas. (b) *In vivo* bioluminescence, imaging showed that exosomes loaded with si-PDGFR*β* had relatively high targeting ability. (c) H&E staining indicated that the si-PDGFR*β*-Exo-treated group induced more necrotic cells than the PBS and Unload-Exo groups. TUNEL assay indicated that si-PDGFR*β*-Exo induced apoptosis. (d) Immunoblot detection demonstrated that si-PDGFR*β*-Exo significantly decreased p-PI3K, p-AKT, EZH2, and PDL1 proteins (^∗∗∗^*P* < 0.001 vs. PBS or Unloaded-Exo group).

**Figure 7:** The evaluation of exosome treatment. (a) Body weight had no statistically difference between Unload-Exo, si-PDGFR*β*-Exo, and PBS groups. (b) The liver, spleen, heart, lung, and kidney functional tests showed no remarkable diversities among three groups. (c) Liver function of the mice in three groups by biochemical blood test showed no significant differences.

**Table 1:** Antibody information of immunoblot.

Antibodies	Dilution rates	Product codes	Manufacturers
*β*-Actin	1 : 1000	PA5-35201	Invitrogen
PDGFR beta	1 : 2000	Ab69506	Abcam
EZH2	1 : 1000	Ab283270	Abcam
p-Akt	1 : 1000	Ab38449	Abcam
Akt	1 : 1000	Ab8805	Abcam
p-PI3K	1 : 1000	Ab278545	Abcam
PI3K	1 : 1000	20584-1-AP	Protein Tech
CD63	1 : 1000	Ab134045	Abcam
TSG101	1 : 1000	Ab125011	Abcam
Bax	1 : 2000	PA5-17216	Invitrogen
Bcl-2	1 : 10000	AM4302	Invitrogen
Cleaved caspase-3	1 : 1000	ab155938	Abcam
Goat anti-mouse IgG H&L (HRP)	1 : 10000	ab6728	Abcam
Goat anti-rabbit IgG H&L (HRP)	1 : 10000	ab6721	Abcam

## Data Availability

The datasets for this study are available from the corresponding author upon reasonable request.

## Supplementary Materials

Supplementary Materials Figure S1: PDGFR*β* was activated in clinical GBM samples. Both bioinformatic analysis and IHC results revealed that PDGFR*β* was up-expressed in tumor tissues of GBM.
